# The Impact of e-Learning Systems on Motivating Students and Enhancing Their Outcomes During COVID-19: A Mixed-Method Approach

**DOI:** 10.3389/fpsyg.2022.874181

**Published:** 2022-07-29

**Authors:** Fethia Yahiaoui, Riad Aichouche, Khalil Chergui, Said Khalfa Mokhtar Brika, Mohmmad Almezher, Adam Ahmed Musa, Imane Ahmed Lamari

**Affiliations:** ^1^University of Oum El Bouaghi, Oum El Bouaghi, Algeria; ^2^University of Bisha, Bisha, Saudi Arabia; ^3^Department of Management Administration, Faculty of Economics, University of White Nile University, Kosti, Sudan

**Keywords:** e-Learning systems, student motivation, student outcomes, COVID-19, mixed-method approach

## Abstract

e-Learning is a key strategy in the course of higher education to improve the results of the educational process and stimulate student motivation. The COVID-19 pandemic imposed on Algerian universities to adopt e-Learning systems to search for effectiveness and efficiency of academic approaches. This paper seeks to remedy these problems by analyzing the impact of e-Learning systems on student motivation and outcomes. A mixed-method approach was used in the data analysis. We conducted the study as a survey, with data being gathered *via* questionnaires distributed to 398 students. The questionnaire includes open questions that were qualitatively analyzed using content analysis with Nvivo, besides Likert scale questions were quantitatively analyzed and modeled using Structural equation modeling (SEM) with Amos to accomplish the path analysis of the research model. The results of the study showed that student motivation (Attention, Relevance, Confidence, and Satisfaction) and student outcomes (knowledge, skills, and attitudes) are significantly affected by e-Learning systems (Technical and electronic requirements, personal requirements, perceived value, and credibility of e-Learning). The key findings are discussed, and they provide recommendations for future research.

## Introduction

e-Learning has become an inevitable strategy for higher education institutions, especially with the emergence of the COVID-19 pandemic, which was imposed different configurations of learning and teaching processes toward focusing more on: blended learning, distance learning, online learning, and smart learning, e.g., Adnan and Anwar (2020), Claps et al. (2020), Çubukçu and Akturk (2020), and Fadillah et al. (2020).

Therefore, several research groups like Almaiah et al. (2020), Al-Okaily et al. (2020), Alqahtani and Rajkhan (2020), Radha et al. (2020), and Shahzad et al. (2020) have been working on the trend of e-Learning to consider the COVID-19 pandemic and its effects. Shahzad et al. (2020) measured the effects of COVID-19 in e-Learning on higher education institution students.

Al-Okaily et al. (2020) extracted the positive effects of e-Learning on student intention to use e-Learning systems during the COVID-19 pandemic. Radha et al. (2020) reflect in their study on the impact of e-Learning, student interest in using e-Learning resources, and their performance, where e-Learning is subject to challenges to achieve its goals (Almaiah et al., 2020). Also, focus on the Critical Success Factors in this pandemic, especially from the managerial perspective (Alqahtani and Rajkhan, 2020).

This provides a solid foundation on which future research can be built, regarding the effects and credibility of e-Learning on higher education and the effectiveness of e-Learning systems in improving student motivation and outcomes. Up to now, several studies have tested these effects (Harandi, 2015; Fryer and Bovee, 2016; Yilmaz, 2017), and confirmed the role of e-Learning in engendering student satisfaction and motivation.

Islam (2011), Saba (2012), and Logan et al. (2021) established the implications of e-Learning systems to facilitate student learning and outcomes. However, recent studies have tested the likely impact of e-Learning on university students during COVID-19 (Alawamleh et al., 2020; Sankar et al., 2020; Wargadinata et al., 2020).

Algerian universities have also turned toward e-Learning as a strategy for developing educational curricula and teaching processes and forming a bet that guarantees the success of education in light of crises similar to the COVID-19 crisis (Guessar, 2020). Research in this area is of great interest and with a very active research community, in Algeria, many researchers were interested in e-Learning issues and their effects on university students before the COVID-19 crisis (Zine El Abiddine, 2013; Aoued, 2016) and during this pandemic (Guessar, 2020; Zermane and Aitouce, 2020).

A closer look at the literature reveals many gaps and shortcomings. Firstly, most Algerian studies in the field of e-Learning have only focused on measuring the general effects of e-Learning, and have not been able to check its effects on student motivation and outcomes; this is what you should focus on (Abou El-Seoud et al., 2014). Secondly, this particular problem (Measuring the effects of e-Learning on student motivation and outcomes) was not sufficiently addressed in light of the COVID-19 pandemic. Finally, previously published studies on this trend are not consistent, most of them focused on measuring general effects, or measuring special effects (student motivation and outcomes), but with a purely quantitative approach (Radha et al., 2020; Soni, 2020).

However, this method of analysis has several limitations; the most important is not determining the potential effects of e-Learning on qualitative variables, especially when we discuss students’ motivation and outcomes (Heller and Sottile, 1996; Saeed and Zyngier, 2012).

The problem of the study is to identify the effects of e-Learning and its contribution to stimulating Algerian students’ motivation and enhancing their educational outcomes during the COVID-19 pandemic, by relying on quantitative and qualitative methods. What is known to researchers as mixed methods? (Johnson et al., 2007; Denzin, 2010; Creswell, 2011).

Then, this major problem includes two sub-problems: The first is to measure the effects of e-Learning on stimulating students’ motivation, like the following previous studies (Barolli et al., 2006; Lanzilotti et al., 2009; Harandi, 2015; Fryer and Bovee, 2016; Govorov et al., 2016; Yilmaz et al., 2017). The second is to determine the effects of e-Learning in enhancing student outcomes, approximating the following prior studies (Islam, 2011; Saba, 2012; Koraneekij and Khlaisang, 2015; Logan et al., 2021).

## Theoretical Background

Many high education institutions have attempted to encourage e-Learning in response to the requirement of educational continuity in light of COVID-19. This raised a question about the feasibility and effectiveness of this process under this circumstance, particularly for universities unfamiliar with this learning style.

Alismaiel (2021) defined e-Learning as a method of learning that is based on formalized education and employs online databases or resources. For Looi (2021), e-Learning is more than making teaching materials digital, it is also associated with various psychological and social factors. In e-Learning, every aspect of the educational process, from implementation to assessment, is aided by technology, including media and learning support tools (Harahap and Fitri, 2021).

Furthermore, the usage of e-Learning enables educators to improve the quality of education by using quick replenishing global educational resources. Also, by increasing the amount of autonomous work required of students while studying the content (Sandybayev, 2020).

The information and communication technology advancements have permitted new learning ways:

- **Technical and electronic requirements:** The technology requirements of e-Learning investigate concerns of technology infrastructure in the e-Learning environment, infrastructure planning, hardware, and software (Pislae-Ngam et al., 2018).
- **Personal requirements:** Implementing e-Learning into a traditional university’s teaching design is a lengthy and challenging process requiring a systematic approach (Sandybayev, 2020). However, due to the Corona epidemic and the circumstances surrounding the forced shutdown, many universities were obliged to transition into e-Learning, to their lack of preparation. Tan (2020) stated that, although the teaching faculty successfully transitioned from traditional teaching techniques to online learning, the consequences were unclear; the majority of the teaching staff were unprepared for online instruction and were compelled to adjust to the transition as a result of the crisis. The personal dimension relates to the extent of training or willingness to use information technology, especially for students. Student perceptions of e-Learning activities *via* computer use are referred to as “learner attitudes.” For instance, when students are not intimidated by the complexity of using computers, will result in more contented and productive learners.
- **The perceived value of e-Learning:** The term “perceived value” in the e-Learning context refers to students’ overall appraisal of the usefulness of learning based on their views of what they receive and what they provide in return (Faqih, 2016). His study also conducted that perceived value elements positively influence students’ intention to adopt and use e-Learning technologies.

This study aims to provide a conceptual theoretical framework based on previous studies and its adoption as a model to be tested in Algerian universities, this model includes three variables: e-Learning, student motivation, and student outcomes.

### e-Learning and Student Motivation

Motivation is a vital aspect of any educational process, especially as it relates to e-Learning. There is no single definition of motivation. Espinar Redondo and Ortega Martín (2015) stated that the existence of such a wide range of concepts demonstrates the difficulty in describing motivation. So, motivation can be defined as what inspires students to dedicate time to a certain task freely. Also, as their attitudes and feelings about the activity, as well as how long they remain committed to the task (Filgona et al., 2020).

According to Keller (2010), the study of motivation is difficult because there are so many motivating ideas, concepts, and theories produced to explain its different elements and the interplay of environmental, cultural, and personal factors. Keller (1983) introduced the ARCS model of four categories (Attention, Relevance, Confidence, and Satisfaction) as a tool quickly understand the main parts of human motivation, especially in learning motivation, and how to stimulate and keep motivation in each of the four areas (Keller, 2010).

The first step in this model is to maintain learners’ curiosity and interest (Attention), the second is to convince the learner that his or her experience is personally meaningful (Relevance), the third step is to convince the learners that they can understand the material and accomplish an activity or a task (Confidence), and the last step is to be sure that learners feel good about what they did or how it worked out (Satisfaction; Keller, 2010). The increasing number of research shows the positive effects of using an effective e-Learning process and student motivation and participation (Herath et al., 2021).

*H1*: There is a direct and significant impact of e-Learning on student motivation in Algerian universities

### e-Learning and Student Outcomes

According to Prøitz (2010), there is considerable debate and ambiguity around the concept of learning outcomes and the widely accepted definition is concentrated on whether learning and its outcomes can and must be expressed in comprehensive, consistent, pre-determined, and quantifiable terms, or open and flexible ones with limited measurement options. For (Maher, 2004) the term “learning outcomes” is about the student behavior changes because of a learning experience. This change can occur in terms of knowledge, skills, and attitudes. It has long been a concern of researchers and educators that learned motivation has a direct correlation to student progress and intended results (Esra and Sevilen, 2021). For instance, a study (Sandybayev, 2020) conducted that e-Learning is more successful than traditional teaching methods in supporting students enrolled in business courses. In their meta-analysis, Cook et al. (2008) claimed that internet-based learning contributes to knowledge acquisition and skill development compared to non-Internet educational approaches. Also, George et al. (2014) found that online Learning seems to be more successful and can cause an improvement in student knowledge, skills, and attitudes.

*H2*: There is a direct and significant impact of e-Learning systems on student outcomes in Algerian universities

### Student Motivation and Student Outcomes

Several studies have found that student motivation has a direct impact on student outcomes. In this regard, the literature claims that there is a correlation between these two variables, and this study backs up that notion (McKenzie and Schweitzer, 2001; Sankaran and Bui, 2001; Fini and Yousefzadeh, 2011; Richardson et al., 2012; Azizoğlu et al., 2015).

*H3*: There is a direct and significant impact of student motivation on student outcomes in Algerian universities

### e-Learning, Student Motivation, and Outcomes

As discussed above, e-Learning has a significant influence on student outcomes. However, this interaction cannot take place unless there is a motivating factor involved. Learner motivation has long been a focus for researchers and educators since it is linked directly to student progress and the expected outcome (Esra and Sevilen, 2021). Numerous studies have demonstrated that increasing student motivation to learn improves their academic performance and outcomes. Therefore, the relationship between e-Learning and student outcomes is mediated by motivation.

*H4*: the relationship between e-Learning and student outcomes is partially mediated by motivation in Algerian universities

### Research Framework

The research framework is shown in Figure 1.

**Figure 1:** Research framework.

## Materials and Methods

To verify the validity of the theoretical framework that links e-Learning systems, Student motivation and student outcomes, we carried out a mixed approach, also known as mixed models, mixed methods and pragmatism (Creswell and Creswell, 2005; Cohen et al., 2017). A combination of analysis advantages of quantitative and qualitative was attained in this approach.

### Quantitative Data and Sample Selection

This study has been conducted to identify the impact of e-Learning Systems on Student Motivation and Outcomes in Algerian universities. The study was conducted in the form of a survey, with data being gathered *via* a structured questionnaire distributed among the students at all levels. The initial sample consisted of 400 students, 398 questionnaires were collected with an estimated response of 99.5%, which is very acceptable, according to Sekaran and Bougie (2019). A snowball sample (non-probability sample) related to network sampling was chosen because of the expected difficulty of obtaining the lists of all Algerian students (Handcock and Gile, 2011).

The questionnaire contained constructs to be measured for quantitative analysis. Construct measurements items were expressed according to a five-point Likert scale that was defined as follows: 1 = strongly disagree, 2 = disagree, 3 = medium agree, 4 = agree, and 5 = strongly agree. The questionnaire included three major constructs in addition to demographic data: e-Learning systems which have three dimensions (Technical and electronic requirements, personal requirements, perceived value of e-Learning, or credibility of e-Learning), Student motivation contains four dimensions [Attention, Relevance, Confidence, and Satisfaction, the ARCS model developed by Keller (1987)], student outcomes which contains three dimensions (Knowledge, Skills, and Attitudes).

Reliability and validity were calculated using Cronbach’s alpha and Guttman split-half, it was performed *via* SPSS software (version 25). Table 1 shows the validity and reliability coefficient of the questionnaire constructs.

**Table 1:** Validity and reliability statistics.

Constructs	Cronbach’s Alpha	Guttman split-half	Number of items	Number of cases
e-Learning systems	0.919	0.828	17	398
Student motivation	0.865	0.646	16	398
Student outcomes	0.924	0.881	12	398
Questionnaire	0.909	0.657	45	398

Table 1 provides the summary statistics for Validity and Reliability; it shows that the reliability coefficients (Cronbach’s Alpha) are 0.919, 0.865, 0.924, and 0.909 for the questionnaire, which is within the acceptable limit according to Bland and Altman (1997). It presents also that the Validity coefficients (Guttman split-half) are 0.828, 0.646, 0.881, and 0.657 for the questionnaire, which is within the allowed range according to Jackson (1979). This indicates that the questionnaire employed in this study is suitable for conducting research and drawing conclusions.

### Qualitative Data

According to Geer (1988), survey researchers frequently use open-ended questions to gauge public opinion, this requiring respondent, either vocally or in writing, to construct and present their answers. Predefined categories of responses are not guided in a particular direction (Züll, 2016). This contributes to obtaining qualitative data for the analysis of quantitative results. Many academics believed that triangulation (multi-method approaches) is typically a strategy for boosting research validity and reliability or evaluating findings (Seale, 1999; Stenbacka, 2001; McMillan and Schumacher, 2010).

The study uses qualitative analysis to gain insights into e-Learning systems, student motivation, and outcomes. Qualitative data were collected from three open-ended questions asked in the questionnaire, first related to e-Learning systems (Are you in accord with the policy of the Algerian Universities for e-Learning? If yes state the reasons, if no mention the reasons also), second about student motivation (Are there clear reasons that motivate or demotivate you to learn, succeed, and achieve your university goals? Is e-Learning considered one of these reasons?). Third about student outcomes (If you want one of the students who achieved satisfactory or unsatisfactory results, please state the reasons? Is e-Learning considered one of these reasons?).

### Methods and Analysis Approaches

#### Quantitative Methods

We have used structural equation modeling (SEM) through IBM SPSS Amos 25 to assess the relationships in the research framework and test the hypothesis. Nachtigall et al. (2003) indicate that the comparison of the model to empirical data is the main feature of SEM. This comparison generates so-called fit statistics, which evaluate the model’s fit with the data. This method or co-variance based structural equation modeling (CB-SEM) requires three conditions (Lowry and Gaskin, 2014). Suitable for confirmatory studies and the model must be precisely delimited between the variables, appropriate for large samples (the study’s sample size is greater than 200, with 398 questionnaires gathered), requires a normal distribution of the data shown in Table 2.

**Table 2:** Tests of normality.

Constructs	Skewness	Kurtosis
e-Learning systems	0.022	−0.231
Student motivation	0.877	0.504
Student outcomes	0.054	−0.322
Questionnaire	0.583	0.350

A significant divergence from normality, according to West et al. (1995), is defined as an absolute skewness value >2, and an absolute kurtosis (proper) value >7. Table 2 shows that all of the research variables’ absolute values are less than 2, for skewness and less than 7 for kurtosis, indicating that the data follow a normal distribution.

#### Qualitative Methods

NVivo is a software program that can be used to save, manage, and analyze qualitative data and open-ended questions (Edwards-Jones, 2014). Visualization techniques (thematic analysis, cluster analysis, and cognitive mapping were used to link three variables: e-Learning systems, student motivation, and student outcomes, to confirm the study model qualitatively and test the degree of its agreement) and thought experiments can also help to clarify what might be useful questions (Jackson and Bazeley, 2019).

## Results of Study

To ensure hypothesis testing and study model the results of the quantitative and qualitative studies are given and compared in this section.

### Descriptive Statistics

The table below illustrates the summary descriptive statistics for the study sample.

Table 3 presents a summary of the study sample’s demographic factors, where it appears that most of the respondents are female (247 with a percentage of 62.1), with an age from 21 to 30 (248 with a percentage of 62.3), and most of them are *Ph.D.* students (246 with a percentage of 61.8). This explains the nature of the sample and the respondents who answered the questionnaire. Diment and Garrett-Jones (2007) confirm that demographic characteristics affect the answers and study variables, whose statistics are presented in Table 4.

**Table 3:** Descriptive statistics of the study sample.

Variables	Categories	Frequency	Percent	Mean	*SD*
Sex	Male	151	37.9		
	Female	247	62.1		
	Total	398	100	1.62	0.486
Age	21–30	248	62.3		
	31–40	138	34.7		
	41–50	12	3		
	Total	398	100	2.41	0.55
Study level	Licence	36	9		
	Master	92	23.1		
	Magister	24	6		
	Doctorat	246	61.8		
	Total	398	100	3.21	1.082

**Table 4:** Descriptive statistics of study variables.

Study variables	Minimum	Maximum	Mean	*SD*
Technical and electronic requirements	1.00	5.00	2.7638	0.77186
Personal requirements	1.00	4.60	2.7025	0.69568
Perceived value of e-Learning	1.00	5.00	2.7119	0.82818
**e-Learning systems**	**1.00**	**4.44**	**2.7261**	**0.68007**
Attention	1.00	5.00	2.6263	0.88379
Relevance	1.00	5.00	2.9133	0.80440
Confidence	1.00	4.75	2.3166	0.66745
Satisfaction	1.25	4.75	1.9221	0.61100
**Student motivation**	**1.19**	**4.69**	**2.4446**	**0.58001**
Knowledge	1.00	4.50	2.7374	0.83991
Skills	1.00	5.00	2.7776	0.96874
Attitudes	1.00	5.00	2.9334	0.87702
**Student outcomes**	**1.00**	**4.83**	**2.8162**	**0.79857**

The bold values are the values of the variables, not the dimensions.

The majority of respondents were inclined to “medium agree” for e-Learning systems (mean = 2.7261) and student outcomes (mean = 2.8162), but “disagree” for student motivation (mean = 2.7261), with a weak dispersion of the three variables based on the SD. This is explained by Algerian universities’ recent embrace of e-Learning systems in response to the COVID-19 pandemic, as well as their lack of emphasis on interactive e-Learning, which boosts student motivation and enhances student outcomes (Abdelouafi, 2020; Zina, 2021).

### Correlation Results

The correlation matrix between study variables and constructs is shown in the table below.

The results of the correlation analysis are set out in Table 5, it appears that all correlation coefficients are significant at 0.01 except for the relationship between knowledge and learning systems which seemed with a weak correlation according to Schober et al. (2018), as they are confined to 0.10–0.39, and this is explained by the dependence of Algerian universities on traditional learning (in-person learning) and the recent integration of the e-Learning systems in a way that greatly affects students motivation and outcomes (Djoudi, 2010; Abdelouafi, 2020; Guemide and Maouche, 2021; Zina, 2021).

**Table 5:** Correlation matrix.

Variables and constructs		Attention	Relevance	Confidence	Satisfaction	Student motivation	Knowledge	Skills	Attitudes	Student outcomes
Technical and electronic requirements	R	0.099^*^	0.116^*^	0.210^**^	0.120^*^	**0.170** ^**^	0.020	0.070	0.059	**0.057**
	Sig	0.048	0.020	0.000	0.017	**0.001**	0.690	0.162	0.241	**0.256**
Personal requirements	R	0.060	0.070	0.168^*^ ^*^	0.077	**0.116** ^*^	−0.021	0.011	0.031	**0.008**
	Sig	0.232	0.161	0.001	0.126	**0.021**	0.672	0.834	0.540	**0.872**
Perceived value of e-Learning	R	0.189^**^	0.098	0.314^**^	0.353^**^	**0.289** ^**^	0.145^**^	0.253^**^	0.188^**^	**0.222** ^**^
	Sig	0.000	0.050	0.000	0.000	**0.000**	0.004	0.000	0.000	**0.000**
**e-Learning systems**	**R**	**0.135** ^**^	**0.108** ^*^	**0.264** ^**^	**0.215** ^**^	**0.221** ^**^	**0.059**	**0.133** ^**^	**0.109** ^*^	**0.114** ^*^
	**Sig**	**0.007**	**0.031**	**0.000**	**0.000**	**0.000**	**0.238**	**0.008**	**0.030**	**0.022**
Knowledge	R	0.184^**^	0.117^*^	0.236^**^	0.197^**^	0.230^**^	1	0.738^**^	0.624^**^	0.878^**^
	Sig	0.000	0.020	0.000	0.000	0.000		0.000	0.000	0.000
Skills	R	0.298^**^	0.197^**^	0.278^**^	0.264^**^	0.331^**^	0.738^**^	1	0.709^**^	0.923^**^
	Sig	0.000	0.000	0.000	0.000	0.000	0.000		0.000	0.000
Attitudes	R	0.186^**^	0.108^*^	0.159^**^	0.131^**^	0.189^**^	0.624^**^	0.709^**^	1	0.872^**^
	Sig	0.000	0.031	0.001	0.009	0.000	0.000	0.000		0.000
**Student outcomes**	**R**	**0.253** ^**^	**0.160** ^**^	**0.253** ^**^	**0.224** ^**^	**0.284** ^**^	**0.878** ^**^	**0.923** ^**^	**0.872** ^**^	**1**
	**Sig**	**0.000**	**0.001**	**0.000**	**0.000**	**0.000**	**0.000**	**0.000**	**0.000**	

** Correlation is significant at the 0.01 level (two-tailed).

* Correlation is significant at the 0.05 level (two-tailed).

The bold values are the values of the variables, not the dimensions.

### SEM Results

Thom (1983) indicates that path analysis is a powerful tool for conceptualizing research and connecting theory to the “real world.” Therefore, this technique was used in our study to find direct and indirect links between variables to test the study’s hypotheses and model in the reality of Algerian universities. The structural model’s outputs are shown in the figure below.

According to Browne and Cudeck (1992), the fit indices of the path model are attained; therefore, the relative chi-square value is less than 5 (3.964), indicating that the suggested model in the study is consistent with the real data. The values of the normed-fit index (0.935), comparative fit index (0.950), and Tucker Lewis index (0.932) are all very close to one, indicating that the study hypothetical model is far from zero (which assumes no relationship between the study variables), as well as a value of RMSEA is 0.086, clearly showing a match between the hypothetical model and the real data. This all leads us to accept the Research framework (Figure 1), as well as the hypotheses which are listed in the table below.

The findings of the entire latent construct are presented in Table 6. The first step is to determine whether our study hypothesis is valid or not. Value of *p* is regarded as significant if it is less than 0.05. The data, in particular, point to rejecting the null hypotheses and accepting the alternative hypotheses (H_2a_, H_2b_, H_3a_, H_3b_, H_3c_, and H_4_), on the other hand, the null hypotheses are accepted and the following alternative hypotheses are rejected (H_1a_, H_1b_, H_1c_, and H_2c_). In this situation, six of the 10 study hypotheses are significant with the acceptance of the study model by looking at the goodness of fit in Figure 2.

**Table 6:** Direct and indirect effects in structural model.

Effect type	Path	Estimate	p-Value	Hypothesis	Results
Direct	e-Learning → Student motivation	0.217	***	H_1_	Supported at 0.01
	e-Learning → Student outcomes	0.083	0.028	H_2_	Supported at 0.05
	Student motivation → Student outcomes	0.217	***	H_3_	Supported at 0.01
Indirect	e-Learning → Student motivation → Student outcomes	0.217*0.217 = 0.047	***	H_4_	Supported at 0.01

***Path is significant at the 0.01 level.

**Figure 2:** Structural model.

In terms of direct effects, personal requirements and the perceived value of e-Learning have a significant impact on student motivation and outcomes, and student motivation has a considerable impact on student outcomes. In terms of indirect effects, the perceived value of e-Learning has a significant impact on enhancing student outcomes through student motivation. On the contrary, we find that technical and electronic requirements have no significant effect on student motivation and outcomes for direct effects and that technical and electronic requirement. In addition, personal requirements have no significant effect on improving student outcomes through student motivation for indirect effects.

### Qualitative Results

According to Braun and Clarke (2006) thematic analysis is a method for describing qualitative data, but it also incorporates interpretation in the processes of selecting codes and creating themes and respondents’ evaluations of Algerian universities’ e-Learning experience through NVivo12 outputs:

Figure 3 provides an overview of respondents’ attitudes regarding e-Learning systems, student motivation, and outcomes in Algerian universities. According to the open-ended questions, there are two trends. Firstly, the positive view; which constituted 52% of the respondents in e-Learning who agree with the policy of the Algerian Universities for e-Learning, and it also constituted 66.33% for the student’s motivation, and the belief that e-Learning is one of the reasons for improving students motivation, and 48.40% for the student’s outcomes among the respondents who supposed that e-Learning was a reason to enhance their outcomes. Secondly, the negative view in which the respondents believe the opposite and prefer in-person learning, which constituted 48% for e-Learning systems, 33.77% for the student motivation, and 51.60% for student outcomes. This is explicated by two features: the importance of e-Learning systems in Algerian universities, and the emphasis on blended learning in improving students’ motivation and results.

**Figure 3:** Matrix query of thematic analysis.

Eden, Jones, and Sims define cognitive mapping as a modeling technique that aims to show ideas, beliefs, values, and attitudes. Their relationships with one another are in a form that is amenable to study and analysis (Northcott, 1996). According to this approach, Figure 4 shows the relationship between the study variables based on the cluster analysis results:

**Figure 4:** Cluster analysis of study variables.

Figure 4 shows that respondents believe there is a clear relationship between e-Learning systems and enhancing student motivation and outcomes. The coefficients of correlation indicated in the table below can be used to estimate this relationship.

Table 7 shows that there is a strong relationship between e-Learning systems and student motivation in the pop-up, with a correlation coefficient of 0.984872, followed by a strong relationship between e-Learning systems and student outcomes in the second degree, with a correlation coefficient of 0.885074, and a strong relationship between the student’s motivation and outcomes in the third degree, with a correlation coefficient of 0.984872, followed by the relationships between other variables that appear with weak to moderate correlation coefficients. This is explained by several aspects: first, there is a strong relationship between the three study variables; second, there is a relationship between the variables and their inverse (for example, talking about motivation leads the interviewer to discuss demotivating); and third, there is a very weak relationship between e-Learning systems and failure to enhance students motivation and outcomes.

**Table 7:** Pearson correlation coefficient.

**Code A**	**Code B**	**Pearson correlation coefficient**
Enhancing student motivation	e-Learning systems	0.984872
Enhancing student outcomes	e-Learning systems	0.885074
Enhancing student outcomes	Enhancing student motivation	0.844271
Failure to enhance student motivation	Enhancing student motivation	0.51375
Failure to enhance student motivation	e-Learning systems	0.497906
Failure to enhance student motivation	Enhancing student outcomes	0.451398
Failure to enhance student outcomes	Failure to enhance student motivation	0.469979
Failure to enhance student outcomes	e-Learning systems	0.399236
Failure to enhance student outcomes	Enhancing student motivation	0.393109
Failure to enhance student outcomes	Enhancing student outcomes	0.372196

## Discussion and Implications

This paper is a modest contribution to the ongoing discussions about the impact of e-Learning systems (technical and electronic requirements, personal requirements, and perceived value of e-Learning) in enhancing student motivation (attention, relevance, confidence, and satisfaction) and student outcomes (knowledge, skills, and attitudes) in Algerian universities. The author’s attention was focused on three major problems, the first of which is the impact of e-Learning systems on student motivation, the second is the impact of e-Learning systems on student outcomes, and the third is the impact of the student’s motivation on their outcomes, using the mixed method, quantitative approach, or path analysis of the data of 398 questionnaires distributed to Algerian university students with Amos, also qualitative analysis of open-ended questions in this survey using NVivo.

The originality of our method arises from the fact that we linked three key elements in Algerian higher education: e-Learning systems, student motivation, and student outcomes, where the relationship between these variables was measured using the mixed method (quantitative and qualitative approaches). The quantitative findings revealed that personal requirements and the perceived value of e-Learning have a significant effect on students’ motivation and outcomes. In addition, to a significant effect on the student’s motivation for their outcomes. On the other hand, there is an indirect significant effect of the perceived value of e-Learning on student outcomes through student motivation. The qualitative findings validated the usefulness of e-Learning systems in motivating the students and increasing their outcomes, especially when used in conjunction with an in-person learning system.

These results concur in good agreement with other studies which studied the three basic problems of this research paper. First, regarding the effect between e-Learning systems and student motivation, at the quantitative level, Rovai et al. (2007) confirmed that e-Learning students had higher intrinsic motivation (to know, do things, and feel stimulation) than on-campus students who attend face-to-face sessions, Abou El-Seoud et al. (2014) emphasized that the usage of interactive components of e-Learning, such as the Moodle e-Learning platform, boosts undergraduate students motivation in Egyptian universities, this is also consistent with the study of Harandi (2015), which confirmed that students are more likely to be motivated when using e-Learning, As for Beluce and Oliveira (2015), through their analysis of the data of 572 students from the Brazilian state of Paraná, they confirmed that for educators and psychologists who work with learning, the data demonstrated considerable rates of autonomous motivational behavior, Goh et al. (2017) analyzed 670 questionnaires distributed to Malaysian universities students using exploratory factor analysis and regression analyses, this research shows how important it is for university administrators and teachers to develop e-Learning courses that maximize student’s motivation. This is in agreement with Sandybayev (2020) who established that the use of an e-Learning approach, particularly in the business school learning environment, as well as the active use of interactive features such as BBL, enhances motivation.

At the qualitative level, there are several studies whose results agree with the results of our study, the most important are: Yang and Cornelius (2004) who asserted that students have a positive experience were found to be flexibility, cost-effectiveness, electronic research availability, simplicity of connection to the Internet, and a well-designed class interface. Shroff et al. (2007) suggested that a pedagogically driven portfolio of learning activities be used, including well-selected and integrated audio, video, and data technologies in global e-Learning situations to enhance student motivation, Gustiani (2020) used thematic analysis of interviews and discovered students motivation for e-Learning was influenced more by their desire to gain new skills and their delight of trying out new learning methods.

All of these investigations back up the conclusion of our research paper, but it is not a widely accepted view. On the one hand, we may discover that the presence of learning affects the student’s motivation; Francis et al. (2019) found that while e-Learning and face-to-face students may differ in academic outcomes, they do not differ in motivation or student characteristics. On the other hand, we find that e-Learning does not stimulate student motivation in some environments and for some students, as confirmed by Esra and Sevilen (2021) who found that students believe e-Learning hurts their motivation due to a lack of social connection, a mismatch between expectations and material, organizational issues, and the organization of the learning environment.

Second, regarding the effect of e-Learning systems on student outcomes, several studies confirmed the findings of our research paper, Eom and Arbaugh (2011) emphasize that student outcomes improve through e-Learning. At the level of quantitative results, using PLS-SEM Islam (2013) confirmed that e-Learning adoption antecedents (ease of use, utility, enjoyment, system quality, information quality, service quality, self-efficacy, usability, and playfulness) have an impact on e-Learning adoption outcomes (learning assistance, community building assistance, and academic performance). Goh et al. (2017) confirmed that e-Learning courses maximize student learning outcomes in Malaysian universities; Ritonga et al. (2020) also concluded that e-Learning has an impact on student learning outcomes. Baber (2020) confirmed that the factors–interaction in the classroom, course structure, instructor knowledge, and facilitation in e-Learning systems are positively influencing students’ perceived learning outcomes.

Other investigations support the findings of our study on a qualitative level concerning the impact of e-Learning on student outcomes. Blackmon and Major (2012) explored that some students were satisfied with their online courses and enrolling in an online program related to their jobs was very beneficial for academic outcomes. The thematic analysis used by … that the access and use of technological resources in classrooms, implementing the e-Learning methodology the COVID-19 lockdown affect the academic performance and student outcomes.

The issue of the consistency of the impact of e-Learning on student outcomes persists. The e-Learning methodology may affect student outcomes if it is used as a pillar of attendance learning. Or what is known as blended learning? This was confirmed by Kintu et al. (2017) who showed that blended learning design features (technology quality, online tools, and face-to-face support) and student characteristics predicted student outcomes. In addition, e-Learning may not affect the results of some students who are not skilled in using them or who do not have the requirements, including an internet connection. This is what was confirmed by Agbejule et al. (2021), who showed that there are several barriers to the success of e-Learning, the most important of which are instructional concerns, lack of social connection, type of educational program, and geographical area.

Finally, multiple investigations have supported the conclusions of our research work about the effect of student motivation on student outcomes. In this regard, this study backs up the literature’s claim that there is a link between motivation and student outcomes (McKenzie and Schweitzer, 2001; Sankaran and Bui, 2001; Fini and Yousefzadeh, 2011; Richardson et al., 2012; Azizoğlu et al., 2015). Numerous studies have demonstrated this relationship using quantitative and qualitative approaches, for quantitative methods, Goodman et al. (2011) established that there is a high association between intrinsic motivation, extrinsic motivation, and academic performance and outcomes using Pearson correlation coefficients for empirical results from 254 commerce faculty students the University of the Western Cape (Ferreira et al., 2011). Also proved that intrinsic motivation positively and significantly influences perceived learning in the course using the structural equation model.

Similarly, Nur’Aini et al. (2020) demonstrated that the learning motivation of students significantly positive impact their learning outcomes using simple linear regression to analyze the data of a sample of 1,125 students.

For qualitative methods, in their qualitative study, Saeed and Zyngier (2012) arrived at several conclusions, the most notable of which is that extrinsic motivation worked to foster ritual engagement in students, but intrinsic motivation aided true student involvement in learning. Students with both levels of motivation engaged in their learning in a variety of ways.

Because of the differences between the students and the academic environment, these results are not always correct. Martens et al. (2004), for example, found that students with high intrinsic motivation did not perform better in class in their studies. In addition, Orhan Özen (2017) found that motivation has a low-level positive effect on student achievement in a meta-analysis of 205 studies. Similarly, Howard et al. (2021) found a link between motivation and poor outcomes. As a result, the study has several research limitations.

The results in this study depend on at least four limitations. First, the study did not evaluate the alterations of the relationship between e-Learning systems, student motivation and outcomes, from one university to another, from the academic environment to another, and from students to others. Also, the variances arising from the differences in the professors’ viewpoints may need a meta-study that collects the results of several studies in different environments. Second, one question still unanswered is whether student motivation and outcomes are more influenced by e-Learning than face-to-face learning or vice versa, or by blended learning, this may need another empirical study. Third, the most important limitation lies in the fact that e-Learning is imposed and inevitable during COVID-19, so the degree of its obligation may affect the outcomes and student motivation, either positively or negatively, this needs to compare to the results before and after the pandemic. Finally, to measure the relationship between the study variables, we may need data from a larger sample, and we may need to use other statistical methods. Especially, the analysis of variance. These limitations are considered future research trends.

## Conclusion

The main objective of this research was to look into the effects of e-Learning systems on motivating Algerian university students and improving their educational outcomes during COVID-19. It focused on the relationship between three key variables: e-Learning systems (technical and electronic requirements, personal requirements, and perceived value of e-Learning), student motivation (attention, relevance, confidence, and satisfaction), and student entrepreneurship (knowledge, skills, and attitudes). The researchers accomplished this objective by analyzing the data from 398 questionnaires issued to Algerian university students to provide a set of quantitative and qualitative outcomes.

Summing up the quantitative results, it can be concluded according to the correlation matrix that there is a positive significant correlation between e-Learning systems and student motivation, and there is a positive significant relationship between student motivation and student outcomes. According to the SEM results or path analysis model, personal requirements and the perceived value of e-Learning have a significant effect on student motivation and outcomes. Also, student motivation has an indirect significant effect on the perceived value of e-Learning on student outcomes.

The qualitative results obtained show that student positive attitudes regarding e-Learning systems are more than negative ones, and this positively affects student motivation and outcomes according to the thematic analysis. Using cognitive mapping, researchers also demonstrated the strong relationship between e-Learning systems, student motivation and student outcomes, and substantially e-Learning systems affecting student motivation and increasing their outcomes, especially when used in conjunction with an in-person learning system.

The studied model is considered very important in Algerian universities, especially in light of their transition to e-Learning during COVID-19, where university administrators, leaders, and policymakers in the Ministry of Higher Education and Scientific Research can benefit from the study findings on several levels, including determining the credibility of e-Learning in terms of motivating students and improving their outcomes. Second, looking for successful e-Learning curricula that raise student motivation to study, and third, looking for ways to improve student motivation before looking for ways to improve their achievements. Professors and students might consider this when looking for ways to improve student results.

Based on the promising findings presented in this paper, work on the remaining issues is continuing and will be presented in future papers. The next stage of our research will be the study of the relationships between e-Learning systems, students motivation, and student outcomes: a meta-analysis. Several other questions remain to be addressed, the differences between the effects of e-Learning and face-to-face learning on student motivation and outcomes, and the effects of blended learning on student motivation and outcomes. More experiments will be needed to verify the impact of COVID-19 obligations on the teaching and learning process and student outcomes.

## Data Availability Statement

The original contributions presented in the study are included in the article/supplementary material; further inquiries can be directed to the corresponding author.

## Author Contributions

Study design, data collection and analysis, and manuscript editing and writing were all conducted by FY, RA, KC, and SB. All authors contributed to the article and approved the submitted version.

## Funding

The study is funded by the General Directorate of Scientific Research and Technological Development, Ministry of Higher Education and Scientific Research, Algeria.

## Conflict of Interest

The authors declare that the research was conducted in the absence of any commercial or financial relationships that could be construed as a potential conflict of interest.

## Publisher’s Note

All claims expressed in this article are solely those of the authors and do not necessarily represent those of their affiliated organizations, or those of the publisher, the editors and the reviewers. Any product that may be evaluated in this article, or claim that may be made by its manufacturer, is not guaranteed or endorsed by the publisher.
